This article has been retracted.

# Mutual Trust Influence on the Correlation between the Quality of Corporate Internal Control and the Accounting Information Quality Using Deep Learning Assessment

**DOI:** 10.1155/2022/8257880

**Published:** 2022-08-29

**Authors:** Ying Zhao

**Affiliations:** School of Accounting, Sias University, Xinzheng, Henan 451100, China

## Abstract

There is a close correlation between internal control and accounting information quality in the process of enterprise management, and this correlation drives the effect of internal control on accounting information quality, thus forming the effect that internal control optimization promotes accounting information quality optimization. This paper firstly gives a brief description of internal control and accounting information quality and then evaluates the correlation between internal control and accounting information quality based on deep learning and proposes a specific modeling method. Through the correlation and promotion of internal control and enterprise accounting information quality, the optimization of enterprise accounting information quality is achieved. And in combination with the actual case analysis, it is found that the method of this paper can achieve 92% accuracy of correlation analysis, and the analysis is more efficient.

## 1. Introduction

At the beginning of the twenty-first century, a series of financial fraud and audit failure cases broke out in the global capital market one after another, such as Enron, WorldCom, and Yinguangxia. In 2019, the Chinese market even broke out the financial fraud cases of Kangmei Pharmaceutical and Kangde Xin one after another [1]. These cases have shocked stockholders while also triggering discussions in the community about the effectiveness of external audit work and reflecting deficiencies in the government's development of accounting standards, the industry's regulation, and companies' internal corporate governance. These deficiencies—lack of internal management mechanism and lack of external supervision mechanism—are the causes of SOEs' surplus management behavior [2], and good internal control and external audit happen to be the means of internal management and external supervision of the company. In July 2002, the Sarbanes-Oxley Act was enacted in the United States to strengthen the regulation of the accounting profession and to improve the accuracy and reliability of corporate disclosures, which emphasized the importance of internal control systems [3]. Since 2008, the Chinese regulatory authorities have promulgated a series of rules and regulations, collectively known as the “One Standard and Three Guidelines,” to strengthen the daily management of enterprises and improve their internal control. These regulations have opened a new period of comprehensive construction of internal control systems for Chinese enterprises [4].

The Audit Office in the “Thirteenth Five-Year Plan national audit work development plan” proposed to promote the vitality of the state-owned economy, to promote enterprise reform, and to achieve full audit coverage of enterprises; the audit objective is to promote the quality and efficiency of enterprises: (1) comprehensive audit of state-owned capital investment and operation companies; (2) at least one audit of state-owned and state-owned capital-dominated enterprises within five years, focusing on the authenticity, integrity, and value preservation and appreciation of state-owned assets within and outside the enterprise, assets, liabilities, profit and loss, major investment decisions and investment performance, development potential and risk potential, corporate governance and internal control of the enterprise, and the compliance with relevant national laws and regulations; (3) paying attention to the implementation of major national policies and measures by enterprises. From this document, it can be seen that the current government audit of enterprise audits focuses on three aspects; one is related to enterprise performance, such as attention to the allocation and operational efficiency of capital and investment performance; the second is related to the quality of accounting information, such as the authenticity and integrity of assets and assets and liabilities profit and loss; the third is related to the internal control of enterprises, such as corporate governance, internal control, and compliance with laws and regulations. The third is related to the internal control of enterprises, such as corporate governance, internal control, and compliance with laws and regulations.

According to the principal-agent theory, the principal, who has the ownership, and the agent, who has the management, have conflicting interests, and the principal cannot fully supervise the agent, and the agent has the motivation and ability to harm the interests of the enterprise for his own benefit, thus giving rise to the principal-agent problem. Among them, information asymmetry is one of the causes of this problem. High quality accounting information in financial reports can effectively alleviate the agency problem caused by information asymmetry. Accounting information, as a carrier of the business status, reflects the efficiency and effectiveness of the business operation. For internal and external stakeholders, they can use the accounting information to understand the real business situation of the enterprise and use it as a basis to make decisions such as investment and disinvestment. Then it is especially important for users of financial statements to obtain a true and reliable financial report.

In the process of obtaining true and reliable financial reports, internal control and external audit of enterprises play an important role. Internal controls aim to provide reasonable assurance that the financial reports provided by the company are true and reliable, and their quality profoundly affects the quality of accounting information of the company. In addition, internal control can also play a key role in preventing fraud, addressing operational risks, and safeguarding the company's property [5].

## 2. Related Work

As an indispensable part of modern corporate governance system, the role of internal control system has been highly recognized in the capital market. Internal control, as a management activity within an enterprise, controls the generation and transmission of accounting information. Theoretically, ensuring the quality of corporate accounting information is one of the core objectives of the internal control system, and effective internal control can improve corporate management, increase efficiency and effectiveness, and improve the quality of corporate accounting information, thus promoting the long-term stable development of the enterprise [6].

According to scholars, internal control is the first line of defense for companies against financial reporting misstatements [7], and safeguarding the truthfulness of corporate accounting information and asset security is the main line of the continuous development of internal control theory, and some even consider the issue of the relevance of internal control effectiveness to the quality of corporate accounting information as the fundamental topic of internal control theory research [8], which is related to the vitality and development direction of internal control.

The following contradictory views on the relationship between internal control and accounting information quality have been found through previous studies. Most foreign scholars take SOX as the research event to explore the changes in the quality of corporate accounting information before and after the implementation of the Act. The SOX Act mandates companies to evaluate and disclose their internal controls by legislation. For example, [9] classifies companies into those with corporate-level internal control deficiencies and those with effective implementation of internal control systems. A controlled study found that companies with internal control deficiencies at the corporate-level exhibited more robust accounting information after the enactment of SOX, but there was no significant difference in the robustness of accounting between companies with internal control deficiencies at the operational level and companies with effective internal controls. For example, [10] studied 4441 companies' financial data before and after the Act and found that companies were more prudent before the implementation of the Act, as evidenced by later recognition of earnings and earlier recognition of losses.

Our scholars [11] and others found that high quality internal control does not imply high quality accounting surplus, the quality of surplus did not improve significantly when firms improved the quality of internal control, and the quality of accounting information did not improve significantly even when firms disclosed internal control evaluation reports in a timely manner. Further, [12] verified whether internal control affects different business relationships differently by classifying firms' business relationships into supplier-relationship type and customer relationship type. They found that the higher the quality of internal control, the less positive the surplus management, and there is no significant change in negative surplus management in the supplier-relationship type of business. In other business relationships, high quality internal controls did not have a significant inhibitory effect on surplus management. Some scholars even found that although high quality internal control inhibits accrual surplus management by executives, it invariably leads to more insidious true surplus management [13].

And most domestic and foreign scholars have found that corporate internal controls significantly and positively affect the quality of accounting information. On the foreign side, scholars' studies have suggested that high quality internal controls can improve the quality of a firm's accruals, improve the robustness of accounting information, and reduce the firm's surplus management [14].

On the domestic side, some scholars point out that the primary factor affecting the quality of accounting information in a firm is the internal control environment [15], but the power structure within the firm affects the relationship between the two [16]. The first is that internal control only exerts an improving effect on accounting information quality when the power of corporate executives is not concentrated; second, if executive power is further divided into structural power, reputational power, political power, and expert power, they find that structural power reduces the inhibitory effect of internal control on surplus management, but expert power and reputational power reinforce that inhibitory effect, while political power has no significant effect. Reference [17] found that the more rational the corporate governance arrangement and the higher the quality of internal control, the higher the quality of accounting information disclosed by the firm, where internal control positively moderates the effect of corporate governance on the improvement of the quality of disclosed accounting information. Reference [18] investigated the relationship between the effectiveness of internal control, firm quality, and the quality of the firm's financial reporting and found that there is a correlation between them. Reference [19] further found that high quality internal control significantly improved the value relevance of accounting surplus, although surplus persistence did not significantly improve when the quality of internal control improved; reference [20] proposed a similar conclusion that higher internal control effectiveness was accompanied by better comparability of accounting information, but the enhancement effect was worse for state-owned firms compared to non-state-owned firms. Literature [21] contradicts the findings of [22], which used 2007–2008 financial accounting data of Chinese A-share listed companies and found that firms without internal control deficiencies have significantly higher robustness of accounting information and accrual quality than those with deficiencies. Similarly, [23] contradicts the findings of [24], where they found that internal control effectiveness is significantly and negatively related to the degree of surplus management activities. Furthermore, [25] pointed out that although internal control can be effective in improving the quality of accounting information of a firm, not all elements, specifically the five elements, exert a significant positive effect on the quality of accounting information of a firm.

## 3. Methodology

### 3.1. Measurements of ICQ

The main evaluation methods of ICQ in academia are divided into three types: first, the results of internal control audit reports issued after audit by firms are used as proxy variables; second, questionnaires are conducted on relevant personnel of enterprises to evaluate whether the internal control of enterprises is properly designed and effectively implemented based on their scores; third, based on the data of relevant information disclosed by listed companies, experts and scholars build their own. Third, according to the information disclosed by listed companies, experts and scholars have established their own index system. First, listed companies may not be willing to disclose internal audit reports, so they cannot evaluate their advantages; on this basis, some scholars believe that nondisclosure is sufficient to prove that there are some defects in internal control, which can be determined by disclosing variables 0–1. Secondly, the questionnaire survey for individual enterprises is suitable for case analysis, but not for empirical analysis of the overall situation.

### 3.2. Measurement of Accounting Information Quality

As mentioned earlier, there are two main models for measuring the quality of accounting information at home and abroad. The first model is to find proxy variables of accounting information quality such as the degree of surplus management; the second model is to use multiple indicators using models to calculate them together.

The accrual principle, which is the basis of accounting measurement for modern enterprises, requires enterprises to account for and measure realized revenues and expenses that should be borne, regardless of whether they are actually received or paid, as revenues and expenses for the current period. Therefore, under this principle, the surplus of an enterprise can be divided into two parts according to whether it is received or paid. One is the net cash flow from operating activities, which measures the portion of earnings that the company can actually capture, while the profits recorded in the form of receivables and thus not actually captured by the company are accrued profits. The accrued profit is divided into a manipulable part and a nonmanipulable part according to whether the company can manipulate it or not. For the former, depending on the risk appetite of the enterprise, the enterprise can choose different accounting policies to manipulate this part; for example, in order to increase the book profit, the enterprise can adjust to reduce the amount of bad debt accrual of accounts receivable and underaccount for the resulting bad debt loss to achieve the purpose of whitewashing the statement. For the nonmanipulable part, it is difficult to be manipulated by enterprises due to the constraints of accounting treatment.

Based on the fact that the quality of accounting information is measured to some extent by the value of manipulable accrued profits accumulated over a certain period of time, then the level of accounting information quality of an enterprise is reflected by the measurement of manipulable accrued profits. The smaller the amount of the manipulable portion, the higher the quality of the enterprise's accounting information. Academics currently measure manipulable accrued profits mainly by using the accrued profit separation method, under which scholars have developed numerous models to measure the degree of corporate surplus management, such as the modified Jones model, the Dechow-Dichev model, and the Lu Jianqiao model. In this paper, the Jones model modified by cross section is used to calculate manipulable accrued profit, which reflects the quality of accounting information of the company. The meanings of each indicator of the cross-sectional Jones model are shown in Table 1.

Firstly, the regression of (1) by industry by year is calculated as *α*_0_, *α*_1_, *α*_2_, and the rest are classified according to the primary industry code. Here manufacturing industry is classified according to the secondary industry code of the SEC, and the rest are classified according to the primary industry code, and the industries with less than 10 classifications are excluded, and then the OLS estimates as *α*_0_, *α*_1_, *α*_2_ are substituted into formula (2) to calculate the nonmanipulable surplus of the enterprise, and then the nonmanipulable surplus is brought into formula (3) to calculate the manipulable surplus of the enterprise, and the absolute value (DA) is taken as a measure of the quality of accounting information; that is, the larger the absolute value, the worse the quality of accounting information.

(1) $$\begin{array}{c} \frac{TA_{i,t}}{ATA_{i,t-1}}=\alpha_{0}\times \frac{1}{ATA_{i,t-1}}+\alpha_{1}\times \frac{\Delta REV_{i,t}}{ATA_{i,t-1}}+\alpha_{2}\times \frac{PPE_{i,t}}{ATA_{i,t-1}}+\varepsilon_{i,t}, \end{array}$$

(2) $$\begin{array}{c} \text{NDA}=a_{0}\times \frac{1}{ATA_{i,t-1}}+a_{1}\times \frac{\Delta REV_{i,t}-\Delta REC_{i,t}}{ATA_{i,t-1}}+a_{2}\times \frac{PPE_{i,t}}{ATA_{i,t-1}}, \end{array}$$

(3) $$\begin{array}{c} \text{Da}=\frac{TA_{i,t}}{ATA_{i,t-1}}-\text{NDA}. \end{array}$$

The correlation between the ICQ and the AIP is very complex, and the situation of “one multifunction” is more common in actual enterprise planning. For a project attribute, it has one main purpose, but at the same time it has several functions and may improve the AIP to different degrees, which makes the correspondence between project attribute investment and AIP difficult to determine. Therefore, based on the historical data of enterprises, this paper takes project attribute investment as the input of NN and AIP improvement as the output of NN and establishes a deep confidence network model to explore the intrinsic connection between enterprise ICQ and AIP.

### 3.3. DBN Model

The DBN model consists of several layers of Restricted Boltzmann Machine (RBM). An RBM contains visible and hidden layers, each layer consists of several neurons, and its structure is shown in Figure 1. In the RBM structure, neurons are interconnected between the visible and hidden layers, but there are no connections between neurons within each layer. The visible layer of the RBM satisfies the Bernoulli distribution or Gaussian distribution, while the hidden layer is the invisible feature detected and satisfies the Bernoulli distribution. The visible and hidden layers are connected by a symmetric weight matrix with probabilities satisfying the Boltzmann distribution.

When *v*_*i*_, *h*_*j*_ are given, the conditional probability distribution is

(4) $$\begin{array}{c} \left\{\begin{array}{c} P\left(h_{j}=1|v;\theta \right)=\sigma \left(\sum_{i=1}^{m}w_{ij}v_{i}+a_{i}\right),\\ P\left(v_{j}=1|h;\theta \right)=\sigma \left(\sum_{j=1}^{n}w_{ij}h_{j}+b_{j}\right), \end{array}\right. \end{array}$$

where *θ*=*w*_*ij*_ is the connection weight between *v*_*i*_ and *h*_*j*_; *a*_*i*_ and *b*_*j*_ are the parameters of the RBM model; *v*_*i*_ is the *i* th neuron of the visible layer, corresponding to the investment of the *i* th item attribute; *h*_*j*_ is the *j* th neuron of the hidden layer; *m*, *n* are the number of neurons in the visible and hidden layers, respectively; *a*_*i*_ and *b*_*j*_ are the unit biases of the visible and hidden layers, respectively.

The visible and hidden layers are independent of each other, and the conditional probability of *h* on *v* is

(5) $$\begin{array}{c} \sigma \left(x\right)=\frac{1}{\left(1+e^{-x}\right)}. \end{array}$$

Given 1 set of defined training sets {*V*^*c*^*|c*{1,2,3 … *c*}}, the training objective is to maximize the log-likelihood function of the established model, and by calculating the gradient of the likelihood function, the weight update formula of the RBM can be obtained.

(6) $$\begin{array}{c} \Delta w_{ij}=\varepsilon \left(E_{\text{data}}\left(v_{i}h_{j}\right)-E_{\text{model}}\left(v_{i}h_{j}\right)\right), \end{array}$$

where *E*_data_ is the expected output of the observation layer, and *E*_model_ is the expected output on the probability distribution of the model.

The DBN model consisting of multiple RBMs stacked bottom-up is shown in Figure 2. This deep confidence network is divided into 2 layers, the bottom DBN pretraining model and the top backpropagation (BP) fine-tuning model, respectively.

### 3.4. Model Training Method

The traditional neural network uses BP algorithm to train the network, but with the increase of the number of hidden layers, the BP algorithm has the problems of gradient being gradually sparse and easy to converge to the local minimum. DBN based on deep learning can better solve the problems of BP algorithm by pretraining and fine-tuning the network parameters, which is divided into the following 2 steps.

#### 3.4.1. Pretraining

Train each layer of the network separately and unsupervised, and use the output of the upper layer as the input of the lower layer to ensure that as much information as possible is retained when the feature vectors are mapped to different feature spaces.

#### 3.4.2. Fine-Tuning

The BP network is set up in the last layer of the DBN to receive the output of the RBM as its input, and the network is trained in a supervised manner to achieve top-down fine-tuning of the parameters.

Each layer of the RBM network can only ensure that the weights within its own layer map optimally to the feature vectors in that layer, so the BP network also propagates the deviation information from the top down to each layer of the RBM, fine-tuning the whole DBN network. The whole training process can be regarded as the initialization of the weights of the deep BP network, thus overcoming the disadvantage of the BP network of randomly selecting the initial values and falling into the local optimum, and the training time and convergence speed are significantly improved.

## 4. Case Study

Taking enterprises as an example, 17 local and municipal enterprises participating in AIP investment from 2018 to 2022 and the real design attributes of data are selected as data input and output models for network parameter training. To verify the authenticity and accuracy of the DBN model, the actual data of 17 local and municipal enterprises in 2022 were used. From the ICQ and AIP enterprise evaluation index system, the neurons are corresponding to 7 different ICQ enterprises. The neurons in the output layer are corresponding to 8 AIP, and the number is 1–8.

### 4.1. DBN Model Parameter Determination

The depth of model structure and parameter research will affect the learning time and prediction error of the model. To optimize the learning effect, variable control method is used to compare and optimize the hidden layer of DBN model. At the same time, the mean absolute error (MAPE) is introduced to evaluate the prediction accuracy of DBN model.

(7) $$\begin{array}{c} \text{MAPE}=\frac{1}{np}\sum_{i=1}^{n}\sum_{j=1}^{p}\left|\frac{y_{ij}-{\hat{y}}_{ij}|}{y_{ij}}\right|\times 100\%. \end{array}$$

From Table 2, when the number of hidden layers is 4, MAPE = 9.1%, and the model has the highest accuracy. As hidden layers increases, the prediction error of the model first increases and then decreases, and “overfitting” occurs. And the number of neurons was selected as shown in Table 3.

From Table 3, when the number of hidden layer neurons is 128, MAPE = 8.2% and the model prediction error is the smallest.

### 4.2. Method Validation

To verify the validity of the DBN-based model, the maximum relative error is introduced, which can be expressed as follows:

(8) $$\begin{array}{c} \Delta A=\max_{j}\left\{\left|\frac{y_{j}-{\hat{y}}_{j}}{y_{j}}\right|\times 100\%,\;j=1,2\ldots p\right\}, \end{array}$$

where Δ*A* is the maximum relative error.

The ICQ in cities A, B, and C in 2022 was selected as input and the AIP value as output. The predicted value of each AIP is obtained by adding the actual value of the previous year's index and the predicted index improvement value, and comparing the deviation between the actual and predicted values, the results are shown in Figures 3–5.

From Figures 3 and 4, the predicted values of AIP for cities A, B, and C under the DBN model are basically consistent with the actual values, and the maximum relative errors are 9.45%, 13.21%, and 11.58%, respectively. The maximum relative error corresponds to the AIP for city B, with actual and predicted values of 23.2% and 26%, respectively, and the absolute error is only 2.8%, which has a small impact on the evaluation results of the enterprises. At the same time, considering the deviation of historical data of enterprises and the variability of development level among municipalities, the accuracy of evaluation results of different municipalities under DBN model varies slightly.

### 4.3. Analysis of Correlation between the ICQ and the AIP

Based on the theoretical analysis of the sensitivity of enterprise ICQ and AIP, the impact of changes in ICQ on the quality of each accounting information is analyzed by taking a city enterprise as an example, and the results are shown in Figures 5 and 6.

The results of Figures 5 and 6 show that, with the improvement of the internal control index of enterprises, the impact on the quality of accounting information is becoming more and more obvious. Therefore, when an enterprise implements internal control, it should select the projects that need to be improved according to the development of the enterprise and carry out targeted management of the projects according to the established ICQ and AIP matching analysis model.

#### 4.3.1. Analysis of the Empirical Results of the Relevance of ICQ and AIP

According to the regression results, the F-value of model 6 equation is 217.3 and the corresponding *P* value is less than the significance level of 0.01, which means that the equation of model 6 is valid. The corresponding *P* value is less than the significance level 0.01, which indicates that the effect of internal control index ICQ on accounting information quality SYN is statistically significant, and furthermore, the coefficient value is 0.067, which means that internal control quality is significantly and positively related to accounting information quality, and the higher the internal control index ICQ, the higher the accounting information quality SYN. As the size of the company LNSIZE and the number of years of establishment OLD increase, the quality of accounting information SYN rises. Hypothesis H1 holds. The correlation analysis is shown in Table 4.

#### 4.3.2. Analysis of the Empirical Results on the Relevance of AIP and AIP

According to the regression results of model 7, the F-value of model 7 equation is 217.3, and the corresponding *P* value is less than the meaningful level of 0.01, indicating that model 7 equation is effective. The VIF value of all variables in the model is less than 10, which can detect the lack of consistency between variables within the validity of the model. ABSDA detected that AIP was negative 4.26 and *P* was less than 0.01. It is worth noting that the experiment is statistically significant, with a value of −7005. And the correlation results are shown in Figure 7.

#### 4.3.3. Analysis of the Empirical Results on the Effect of AIP as a Mediating Variable on Internal Control and AIP

The above model test shows that the F-value of model 8 equation is 210.6, which corresponds to a *P* value significantly lower than 0.01, which means that the hypothesis of the model is valid. The adjusted R-squared is 0.373, which indicates that the model 8 hypothesis also actually exists. The corresponding *P* value is less than 0.01, which means that the intermediate ABSDA variable has a very significant impact on the overall development of AIP and also means that the intermediate ABSDA variable has a significant impact on AIP syn. At the same time, model 8 notes that the internal control level of ICQ is quite high, indicating that this intermediate effect is completely indirect. The regression results are shown in Table 5.

## 5. Conclusion

The discussion on the quality of accounting information from the perspective of internal control is an important strategic planning issue and management planning direction for the economy and enterprises at a certain stage of development. From the perspective of internal control, the optimization of enterprise accounting information quality can be carried out as follows: optimization of internal control system and governance structure, optimization of internal accounting control system and accounting function, optimization of personnel control, etc. In the face of the ever-changing market economy, the optimization of accounting information quality with good internal control planning is an important way to realize enterprise efficiency and management innovation.

## Figures and Tables

**Figure 1:** RBM model.

**Figure 2:** DBN-based model for analyzing the correlation between the ICQ and the AIP.

**Figure 3:** Comparison of actual and predicted values of the AIP in city A.

**Figure 4:** Comparison of actual and predicted values of AIP in city B.

**Figure 5:** The impact of changes in the ICQ on each positive AIP indicators.

**Figure 6:** The impact of changes in the ICQ on each negative AIP indicators.

**Figure 7:** Correlation results of different indictors.

**Table 1:** Meaning of each index of the cross-sectional Jones model.

Variable symbol	Chinese name
*TA*_*i*,*t*_/*ATA*_*i*,*t*_	Average total assets
*TA*_*i*,*t*_	Accrued profit
Δ*REV*_*i*,*t*_	Change in operating income
Δ*REC*_*i*,*t*_	Change in accounts receivable
*PPE*_*i*,*t*_	Fixed assets

**Table 2:** Effect of #hidden layers on the accuracy of the model.

Hidden layers	MAPE (%)	Training time (s)
2	11.2	55
3	10.4	176
4	9.2	789
5	9.6	439
6	10.8	608
7	12.4	701

**Table 3:** Effect of #neurons in the hidden layer on the accuracy of the model.

Number of hidden layers	MAPE (%)	Training time (s)
32	10.5	32
64	9.2	286
128	8.1	988
256	9.6	2047
512	10.5	7072

**Table 4:** Correlation analysis.

	SYN	ABSDA	ICQ	LEV	INSIZE	MB	TOP1	INST	OLD
SYN	1	−0.042 ^*∗∗*^	0.041 ^*∗∗*^	0.046 ^*∗∗*^	0.155 ^*∗∗*^	−0.105 ^*∗∗*^	0.015	0.056 ^*∗∗*^	0.082 ^*∗∗*^
ABSDA	−0.042 ^*∗∗*^	1	0.025 ^*∗∗*^	0.074 ^*∗∗*^	−0.033 ^*∗∗*^	0.072 ^*∗∗*^	−0.023 ^*∗∗*^	−0.062 ^*∗∗*^	0.034 ^*∗∗*^
ICQ	0.041 ^*∗∗*^	0.025 ^*∗∗*^	1	0.022 ^*∗∗*^	0.205 ^*∗∗*^	−0.047 ^*∗∗*^	0.103 ^*∗∗*^	0.148 ^*∗∗*^	−0.018 ^*∗∗*^
LEV	0.045 ^*∗∗*^	0.072 ^*∗∗*^	0.024 ^*∗∗*^	1	0.532 ^*∗∗*^	−0.413 ^*∗∗*^	0.108 ^*∗∗*^	0.213 ^*∗∗*^	0.145 ^*∗∗*^
INSIZE	0.155 ^*∗∗*^	−0.033 ^*∗∗*^	0.205 ^*∗∗*^	0.532 ^*∗∗*^	1	−0.539 ^*∗∗*^	0.255 ^*∗∗*^	0.427 ^*∗∗*^	0.099 ^*∗∗*^
MB	−0.106 ^*∗∗*^	0.072 ^*∗∗*^	−0.045 ^*∗∗*^	−0.413 ^*∗∗*^	−0.537 ^*∗∗*^	1	−0.088 ^*∗∗*^	−0.152 ^*∗∗*^	−0.096 ^*∗∗*^
TOP1	0.015	−0.023 ^*∗∗*^	0.101 ^*∗∗*^	0.108 ^*∗∗*^	0.255 ^*∗∗*^	−0.088 ^*∗∗*^	1	0.505 ^*∗∗*^	−0.065 ^*∗∗*^
INST	0.056 ^*∗∗*^	−0.062 ^*∗∗*^	0.148 ^*∗∗*^	0.211 ^*∗∗*^	0.425 ^*∗∗*^	−0.152 ^*∗∗*^	0.505 ^*∗∗*^	1	0.082 ^*∗∗*^
OLD	0.082 ^*∗∗*^	0.036 ^*∗∗*^	−0.018	0.145 ^*∗∗*^	0.099 ^*∗∗*^	−0.094 ^*∗∗*^	−0.065 ^*∗∗*^	0.082 ^*∗∗*^	1

^*∗∗*^ Correlation is significant at the 0.01 level (2-tailed).

**Table 5:** Regression results.

	Hypothesis 1	Hypothesis 2	Hypothesis 3
	SYN	SYN	SYN
ICQ	0.068 ^*∗∗∗*^		0.071 ^*∗∗∗*^
	(4.15)		(4.35)
LEV	−0.472 ^*∗∗∗*^	−0.472 ^*∗∗∗*^	−0.442 ^*∗∗∗*^
	(−6.66)	(−6.65)	(−6.20)
LNSIZE	0.065 ^*∗∗∗*^	0.075 ^*∗∗∗*^	0.064 ^*∗∗∗*^
	(5.12)	(5.99)	(4.98)
MB	−0.097 ^*∗∗∗*^	−0.092 ^*∗∗∗*^	−0.095 ^*∗∗∗*^
	(−15.02)	(−14.48)	(−14.67)
TOP1	0.111	0.125	0.116
	(1.25)	(1.38)	(1.33)
INST	−0.166 ^*∗∗∗*^	−0.168 ^*∗∗∗*^	−0.183 ^*∗∗∗*^
	(−2.65)	(−2.68)	(−2.92)
OLD	0.006 ^*∗∗∗*^	0.006 ^*∗∗∗*^	0.006 ^*∗∗∗*^
	(3.08)	(3.04)	(3.12)
ABSDA		−0.705 ^*∗∗∗*^	−0.735 ^*∗∗∗*^
		(−4.26)	(−4.47)
CONS	−2.546 ^*∗∗∗*^	−2.281 ^*∗∗∗*^	−2.489 ^*∗∗∗*^
	(−8.68)	(−7.87)	(−8.46)
*R* ^2^	0.376	0.376	0.377
ADJ *R*^2^	0.372	0.372	0.373
*F*	217.5 ^*∗∗∗*^	274.5 ^*∗∗∗*^	210.6 ^*∗∗∗*^

## Data Availability

The experimental data used to support the findings of this study can be obtained from the corresponding author upon request.
